The article "Efficacy, Safety, and Impact on Patient Survival of PDL1/PD-1 Inhibitors versus FOLFIRINOX Regimens for Advanced Pancreatic Cancer" was retracted in 2023. Reasons: unreliable results or conclusions; lack of ethics approval or compliance; concerns about the data; concerns about the peer review.

# Efficacy, Safety, and Impact on Patient Survival of PDL1/PD-1 Inhibitors versus FOLFIRINOX Regimens for Advanced Pancreatic Cancer

**DOI:** 10.1155/2022/5430720

**Published:** 2022-06-18

**Authors:** Lang Zhou, Zhaoshu Wu, Chunping Jiang, Shiming Dai

**Affiliations:** ^1^Nanjing University of Chinese Medicine, Nanjing, 210023 Jiangsu Province, China; ^2^Department of General Surgery, Nanjing Hospital of Chinese Medicine Nanjing, 210012 Jiangsu Province, China; ^3^Department of Hepatobiliary Surgery, Nanjing Drum Tower Hospital, The Affiliated Hospital of Nanjing University, Nanjing, 210008 Jiangsu Province, China

## Abstract

**Background:**

Over the last few years, the role of PDL1/PD-1 in pancreatic cancer development has received increasing attention, and this article is aimed at opening up new ideas for the medicine-based treatment of pancreatic cancer.

**Aims:**

To investigate the efficacy and safety of PDL1/PD-1 inhibitors versus FOLFIRINOX regimen in the treatment of advanced pancreatic cancer and its impact on patient survival and to provide a reference basis for clinical treatment of pancreatic cancer.

**Materials and Methods:**

The 116 pancreatic cancer patients treated in our hospital from September 2019 to September 2021 were selected and divided into 58 cases each in the (instance of watching, noticing, or making a statement) group and the comparison group according to the method based on random number table. The comparison group was treated with FOLFIRINOX, and the group was treated with PDL1/PD-1 stopper. The effectiveness, safety, and hit/effect on survival of the patients in the two groups were compared.

**Results:**

The median chemotherapy cycle for all patients was 4 (1-6), and the combined objective remission rate (0RR) was 36% and the disease control rate (DCR) was 80% after no chemotherapy in 116 patients, with 37.5% 0RR and 81.3% DCR in the observation group and 33.3% 0RR and 77.8% DCR in the comparison group. The greatest number of all patients reached SD, 44%; in the observation group, 43.8%; and in the comparison group, 44.5%. The rate of adverse reactions such as hematological toxicity, neutropenia, anemia, thrombocytopenia, nonhematological toxicity, vomiting, fatigue, infection, diarrhea, intestinal obstruction, and peripheral neuropathy was lower in 10.3% of patients in the observation group than in 25.8% of patients in the comparison group, which was significantly different by *χ*^2^ test (*P* < 0.05). The median progression-free survival curve of the two groups was 19 months in the comparison group and 22 months in the observation group. The progression-free survival in the observation group was significantly higher than that in the comparison group, and there was a statistically significant difference between the two groups (*P* < 0.05).

The article "Efficacy, Safety, and Impact on Patient Survival of PDL1/PD-1 Inhibitors versus FOLFIRINOX Regimens for Advanced Pancreatic Cancer" was retracted in 2023. Reasons: unreliable results or conclusions; lack of ethics approval or compliance; concerns about the data; concerns about the peer review.

**Conclusion:**

PDL1/PD-1 inhibitors in combination with FOLFIRINOX regimens have shown longer survival than treatment with FOLFIRINOX regimens for pancreatic cancer patients, with reliable clinical efficacy, tolerable adverse effects, and a high safety profile for patients.

## 1. Introduction

Pancreatic cancer is a highly aggressive, difficult-to-treat, and highly lethal malignancy. About 15% of patients can undergo radical surgery, and most die due to metastasis or recurrence of the tumor, with an overall 5-year survival rate of only 7% [1]. In the last 30 years, despite significant advances in surgery, radiotherapy, chemotherapy, or combination therapy, the prognosis and overall mortality of pancreatic cancer patients have not changed significantly [2]. Pancreatic cancer is a highly aggressive and lethal malignancy with difficult early diagnosis, short median patient survival and poor prognosis [3]. Programmed death ligand-l (PD-Ll) is a member of the B7 family with negative immunomodulatory effects discovered over the last few years, a negative law-based effect on the unable to be harmed response upon binding to its receptor programmed death receptor-l (PD-l) [4]. The differential distribution of PD-1 and PD-L1 in and (containing cancer) tissues provides a new approach to immunotherapy of harmful tumors, and anti-PD-L1/PD-1 disease-fighters have been used in the treatment of tumors to bring significant results [5]. Based on this, this study was conducted to explore the efficacy, safety, and impact on patient survival of PDL1/PD-1 inhibitors and FOLFIRINOX regimen for the treatment of advanced pancreatic cancer, and the findings are now reported as follows.

## 2. Material and Methods

### 2.1. Research Object

Patients gave informed consent before enrollment, communicated fully with patients before the experiment, introduced the content and process of the experiment, related risks and possible adverse reactions, signed the informed consent form after obtaining patients' consent, and informed patients of the test results in strict accordance with the standard operation of the experimental procedure. In this study, the regression of solid tumors was calculated according to the sample size of the cross-sectional survey: *n* = ta2*PQ*/*d*2, where *n* was the sample size, *P* was the incidence of advanced pancreatic cancer, *Q* = 1 − *P*, *d* was the allowable error, *a* = 0.05, and ta = 1.96. The minimum sample size brought into the formula is 95 cases. We actually included 116 patients with PC in a retrospective study, divided into an observation group and a comparison group of 58 cases each according to the random number table method. All included patients were able to receive the PDL1/PD-1 inhibitor or FOLFIRINOX regimen in our hospital after assessment of their medical condition and physical condition by a team of professional physicians.

The article "Efficacy, Safety, and Impact on Patient Survival of PDL1/PD-1 Inhibitors versus FOLFIRINOX Regimens for Advanced Pancreatic Cancer" was retracted in 2023. Reasons: unreliable results or conclusions; lack of ethics approval or compliance; concerns about the data; concerns about the peer review.

### 2.2. Exclusion Criteria

The following are the inclusion criteria: (i) all patients were confirmed to have pancreatic ductal adenocarcinoma by pathology (ultrasound endoscopic puncture, laparoscopic biopsy of metastatic lymph nodes or nodal foci, ascite exfoliative cytology, etc.) according to the Clinical practice guidelines in Oncology [5], or the diagnosis could not be confirmed histologically due to failed puncture, etc., and the clinical diagnosis was made by a surgeon in collaboration with an impacted physician diagnosis of pancreatic cancer; (ii) all patients are in good physical condition, with no organ (harmful, angry behaviors) such as liver or and an Eastern Cooperative Cancer-related medical care Group score (ECOG) of 0 or 1 before (using powerful drugs to help cure disease); (iii) at least 1 measurable deadly and (able to do something well/very good) blood, liver and kidney-related function. Patients with prior adjuvant therapy (including adjuvant radiotherapy or chemotherapy for >4 weeks) and postoperative relapse were eligible for inclusion in this study, and the clinical profile of the selected patients was complete.

The following are the exclusion criteria: (i) age 76 years or older, harmful tumors of the pancreas other than dangerous tumor, history of other types of cancer, and history of drug (strong, bad body reaction); (ii) active and uncontrollable medical disease such as extreme infection and shock, nerve disease > grade2, history of pain-relieving radiotherapy/immunotherapy, and/or lactating women; (iii) neuroendocrine carcinoma or other malignant pancreatic tumors other than pancreatic ductal epithelium, concurrent heterologous tumors at other sites, those who fail to evaluate the efficacy in time during chemotherapy, and those who abandon treatment in the middle of the course due to social factors.

### 2.3. Methods

The control group was treated with the FOLFIRINOX regimen; i.e., oxaliplatin 68 mg/m, irinotecan 135 mg/m, and calcium folinic acid 400 mg/m were given intravenously on the first day of each course, and fluorouracil 400 mg/m was given intravenously by push, followed by fluorouracil 2400 mg/m by continuous intravenous infusion for 46 hours, repeated every 2 weeks, and every 2 courses of treatment were 1 cycle, and the treatment lasted for 6. The treatment lasted for 6 weeks. Additional treatment was administered according to the patient's postchemotherapy status, and the treatment regimen could be changed halfway if chemotherapy was ineffective or intolerable. Before each course of chemotherapy, liver and kidney function and tumor indexes were examined, and chest X-ray and electrocardiogram were completed. Every two cycles, whole abdomen enhanced thin layer CT with 3D reconstruction was performed to evaluate the tumor metastases and the relationship with surrounding large blood vessels, so as to accurately determine whether the treatment could be converted to surgery. During chemotherapy, adjuvant treatments such as gastric protection and antiemetic and nutritional support were provided, and the side effects of chemotherapy were closely followed up for timely management. Patients with biliary obstruction symptoms before or during treatment should be actively relieved by percutaneous transhepatic bile duct drainage (PTCD), endoscopic biliary stent placement, etc., and then chemotherapy should be administered when the patient's physical condition improves. Those with poor general physical condition should be given active improvement of nutritional status before chemotherapy, including intravenous nutritional support, albumin infusion, and diet therapy. PDL1/PD-1 inhibitor therapy was implemented in the observation group; i.e., the observation group was treated with PDL1/PD-1 inhibitors on the basis of the comparison group, i.e., pabrolizumab injection 200 mg, carrilizumab injection 200 mg, sindilizumab injection 200 mg, and treprolizumab 240 mg, which were administered intravenously for 1 h, once every 2 weeks until the patients developed intolerance or disease progression. All patients were given appropriate symptomatic treatment in case of adverse reactions.

The article "Efficacy, Safety, and Impact on Patient Survival of PDL1/PD-1 Inhibitors versus FOLFIRINOX Regimens for Advanced Pancreatic Cancer" was retracted in 2023. Reasons: unreliable results or conclusions; lack of ethics approval or compliance; concerns about the data; concerns about the peer review.

### 2.4. Observation Indicators

All blood samples were taken from 6 ml of venous blood from the elbow on an empty stomach in the early morning of the patient after the intervention, of which 2 ml was used for routine blood tests and the remaining 4 ml was centrifuged at high speed and stored in a refrigerator at 2-80°C. The upper serum was taken after centrifugation at 3000*r* for 10 minutes and kept in an environment of -70°C. Serum markers were measured using the intact-serum marker 10-8000 kit ELISA method from DLS, Sekiguni, using the Burroughs 550 analyser, USA. The PS score was based on the activity status scale developed by the Eastern Cooperative Oncology Group (ECOG) [6] PS score: 0—has the ability to perform completely normal activities with no significant difference from before the onset of the disease; 1—can perform daily activities and tolerate light physical activities but not heavier physical activities; 2—can get up and move around on his own for more than half of the day and can take care of himself and cannot tolerate physical; 3—only partially self-care, with more than half of the day in bed or in a wheelchair; 4—bedridden and unable to manage daily life; and 5—death. The following is the clinical outcome: efficacy is assessed according to the Criteria for Evaluation of the Efficacy of Solid Tumours (RECIST 1.1) [7] and is classified as complete (temporarily free of disease) (CR), partial (temporarily free of disease) (PR), stable (SD), and progressive (PD). In CR, all targets (damage to body parts) disappear, and the short axis value of any disease-related whether or not it is a target must be less than 10 mm. In PR, the sum of the critical radii is used as a reference. In SD, there is a reduction of at least 30% in the sum of the radii of all target by reference to the minimum of the sum of the studied radii of target. In neither PR nor PD, there is an increase of at least 20% in the sum of the radii of all target by reference to the minimum of the sum of the studied (radii of target including cases where the minimum is equal to the critical value), in addition to a complete and total increase in the sum of the radii (note: the presence of a new (damage to a body part) can also be thought about/believed as development or increase over time/series of events or things). The objective remission rate (ORR) is defined as CR + PR and the disease control rate (DCR) as CR + PR + SD. The above indicators were recorded separately. The final assessment objective is the median overall survival time (OS) of the patient. OS is the time from when the patient received the modified regimen chemotherapy to when the patient died.

### 2.5. Statistical Analysis

Repeated measure analysis of variance between groups was used to measure the measurement expressed as the mean ± standard deviation (*X* ± *S*). Count data expressed as a percentage (%) were tested by *χ*^2^. Univariate and logistic multivariate regression analysis was used to compare the influencing factors, and the risk factors with significant differences were screened. The included data that did not conform to a normal distribution were described by *M*(QR), using the Mann–Whitney test. All statistical tests were two-sided probability tests. The statistical significance was *P* < 0.05.

## 3. Results

### 3.1. Comparison of General Information

The comparison of general data such as gender, mean age, basal metabolism, weight, and height between the two groups was not significantly different (*P* > 0.05). See Table 1.

### 3.2. Comparison of Serum Markers

After measuring CA15-3, CYFRA21-1 and CEA in the observation group were significantly lower than those in the reference group, and the differences were all statistically significant (*P* < 0.05), while CAI25 and TPS in the observation group were not significantly different from those in the reference group, and the differences were not statistically significant (*P* > 0.05). See Figure 1.

The article "Efficacy, Safety, and Impact on Patient Survival of PDL1/PD-1 Inhibitors versus FOLFIRINOX Regimens for Advanced Pancreatic Cancer" was retracted in 2023. Reasons: unreliable results or conclusions; lack of ethics approval or compliance; concerns about the data; concerns about the peer review.

### 3.3. Comparison of Clinical Efficacy

The comprehensive objective response rate (ORR) of the 116 patients without chemotherapy was 36%, and the disease control rate (DCR) was 80%. The ORR of the observation group was 37.5%, and the DCR was 81.3%. The ORR of the control group was 33.3%, and the DCR was 77.8%. Among all the patients, SD was the most, accounting for 44%, 43.8% in the observation group, and 44.5% in the control group. See Figure 2.

### 3.4. Adverse Reaction Comparison

The adverse reaction rate of hematological toxicity, neutropenia, anemia, thrombocytopenia, nonhematological toxicity, vomiting, fatigue, infection, diarrhea, intestinal obstruction, peripheral neuropathy, etc. in the observation group was 10.3% lower than that in the control group, which was 25.8%, with significant difference after *χ*^2^ test (*P* < 0.05). See Figure 3.

### 3.5. Survival Analysis

The median progression-free survival was 19 months in the comparison group and 22 months in the observation group. The progression-free survival in the observation group was significantly higher than that in the comparison group, and there was a statistically significant difference between the two. See Figure 4.

## 4. Discussion

PD-1 and PD-L1 belong to the CD28 immunoglobulin superfamily and B7 superfamily, respectively, and PD-1 inhibits the overactivation of the immune response and promotes immune resistance to self-antigens. 2PD-1 is expressed on the surface of various immune cells. In vivo, it is activated by its ligands PD-L1 or PD-L2 [8]. PD-L1 is expressed by various cell types such as immune cells and tumor cells after interacting with cytokines such as interferon- (IFN-) Y. Following interaction with cytokines such as interferon- (IFN-) Y, the PD-1/PD-L1 pathway by various cell types, including immune and tumor cells, maintains immune system homeostasis in vivo and infects it or inflammation [9]. Expression of PD-L1 on the surface of tumor cells is induced by activation of oncogenes and antitumor cytokines [10]. The mitogen-activated protein kinase (MAPK) pathway, PI3K/Akt pathway, and signaling and transcriptional activator 3 (STAT3) have all been shown to bind to the PD-L1 promoter and regulate its transcription [11]. It induces PD-L1 expression on the surface of tumor cells, which in turn induces PD-1 expression on the surface of T cells [12]. The interaction between PD-L1 and PD-1 weakens lymphocyte activation, promotes regulatory T cell function and development, impairs the immune response of antitumor T cells, and prevents tumor cell immune avoidance [13]. Therefore, tumor cells can silence the immune system via the PD-1/PD-L1 pathway, and blocking PD-1/PD-L1 effectively enhances the antitumor activity of immune cells and provides an immune response. It can be enhanced [14]. In recent years, anti-PD-1/PD-L1 therapy has achieved better clinical efficacy in melanoma, renal cell carcinoma, non-small-cell lung cancer, and other tumors and is effective in the largest pathway of advanced and metastatic tumors. It reduces the number of cancers, promotes their metastasis, improves patient survival, and has long-term effects on a wide range of cancer types, especially solid tumors [15].

The article "Efficacy, Safety, and Impact on Patient Survival of PDL1/PD-1 Inhibitors versus FOLFIRINOX Regimens for Advanced Pancreatic Cancer" was retracted in 2023. Reasons: unreliable results or conclusions; lack of ethics approval or compliance; concerns about the data; concerns about the peer review.

In this study, CA15-3, CYFRA21-1, and CEA in the observation group were measured to be significantly lower than those in the reference group, and the comparative differences were all statistically significant. The specific reasons for this are as follows: studies have shown that downregulation of PD-L1 can reduce radioresistance by promoting apoptosis, the combination of radiotherapy and anti-PD-L1 antibody in mouse models synergistically improves antitumor immunity by promoting CD8+ T cell infiltration and reducing the accumulation of MDSCs and tumor-infiltrating regulatory T cells and PD-L1 can be maintained through phosphorylation of OCT4 and Nanog stemness of breast cancer cells [16]. The choice of a single anti-PD-L1 treatment for pancreatic cancer lacks immune response, so it is crucial to overcome the immunosuppressive environment of pancreatic cancer against PD-L1-targeted immunotherapy and enhance immunotherapy activity [17]. Combination therapy with other therapies such as chemotherapy and cancer vaccines can turn tumor cells from “cold” to “hot,” i.e., from nonimmune to immune, and thus sensitive to immunotherapy [18].

The combined objective remission rate (0RR) after chemotherapy-free was 36%, and the disease control rate (DCR) was 80% in 116 patients in this study, with 37.5% 0RR and 81.3% DCR in the observation group and 33.3% 0RR and 77.8% DCR in the comparison group. The greatest number of all patients reached SD, 44%; in the observation group, 43.8%; and in the comparison group, 44.5%. The specific reasons for this are as follows: although there is no consensus on the effectiveness of neoadjuvant chemotherapy or translational therapy for patient treatment, data from studies at several healthcare institutions suggest that the use of PD-1/PD-L1 inhibitors provides better surgical RO resection rates and prognosis [19]. Data from a US study [20] showed that after chemotherapy with a PD-1/PD-L1 inhibitor regimen in 25 patients in the observation group, 11 patients (44%) completed surgical resection, with an R0 resection rate of 86.4% and no perioperative deaths, and a median PFS of 18 months was found for those who completed surgery compared to 8 months for those who did not, significantly prolonging progression-free survival. In a meta-analysis [21], it was observed that of the 12 studies included, 91 patients (28%) of the 325 patients in the observation group completed surgical resection after treatment with PD-1/PD-L1 inhibitors, for an R0 resection rate of 74%. In the current study, the LAP°C patients had a surgical conversion rate of 25% and an R0 resection rate of 75%, a slightly lower surgical conversion rate and a comparable R0 resection rate than the above studies. Survival was 12 months, except for one patient who had died, and the remaining patients were currently alive at 14 months, 22 months, and 10 months. Although this study does not yet demonstrate a significant survival benefit in the observation group over nonsurgical patients due to insufficient sample size data, the PD-1/PD-L1 inhibitor does provide an opportunity for surgical resection in the observation group, which will be further demonstrated as the sample size increases.

The article "Efficacy, Safety, and Impact on Patient Survival of PDL1/PD-1 Inhibitors versus FOLFIRINOX Regimens for Advanced Pancreatic Cancer" was retracted in 2023. Reasons: unreliable results or conclusions; lack of ethics approval or compliance; concerns about the data; concerns about the peer review.

In this study, the rate of adverse reactions such as hematological toxicity, neutropenia, anemia, thrombocytopenia, nonhematological toxicity, vomiting, fatigue, infection, diarrhea, intestinal obstruction, and peripheral neuropathy was 10.3% lower in the observation group than in the comparison group at 25.8%, which was tested to be significantly different. In the comparison group, the most common hematological index was neutropenia much lower than the original regimen, which lies in the active monitoring of patients' hematological indexes before and after chemotherapy and timely whitening treatment, including carrying diethylstilbestrol tablets at discharge to maintain granulocyte levels not only to prevent the risk of infection and other risks but also to prevent patients from delaying chemotherapy due to low granulocyte levels [22]. No thrombocytopenia was observed, while anemia was slightly higher than in the original regimen [23]. Nonhematological indicators lie in the prophylactic use of antiemetic drugs during chemotherapy, including azathioprine and gastrofacial, and the absence of diarrhea and peripheral neuropathy, possibly associated with lower doses of oxaliplatin and irinotecan [24–27].

PDL1/PD-1 inhibitor therapy has opened the door to also play a broad role in immune homeostasis, inflammation, chronic infection, and cancer treatment through multiple pathways [28]. However, several problems remain in the treatment of pancreatic cancer: more than half of patients do not respond to PDL1/PD-1 inhibitor blockade therapy, and there are no current biological markers to distinguish responders from nonresponders [29]. Although the findings of the PDL1/PD-1 inhibitor immune checkpoint pathway have been applied in the management of many patients, most patients have had little response to anti-PDL1/PD-1 inhibitor immunosuppression alone [30]. Thus, PDL1/PD-1 inhibitor immunotherapy has become the basis for combination therapy aimed at increasing the number of patients who respond, but the optimal combination regimen to improve efficacy is unclear [31]. Some patients have experienced autoimmune reactions while applying immunosuppressive agents to treat their tumors, and there is no clear combination regimen to reduce immune-related adverse effects while improving antitumor outcomes. The cost of immunosuppressive therapy is high, and the medical costs are relatively heavy. Therefore, the use of PDL1/PD-1 inhibitors in the treatment of pancreatic cancer requires extensive prospective studies to determine the optimal combination of therapeutic regimens and to develop new directions for the clinical management of pancreatic cancer.

The article "Efficacy, Safety, and Impact on Patient Survival of PDL1/PD-1 Inhibitors versus FOLFIRINOX Regimens for Advanced Pancreatic Cancer" was retracted in 2023. Reasons: unreliable results or conclusions; lack of ethics approval or compliance; concerns about the data; concerns about the peer review.

In summary, the combination of PDL1/PD-1 inhibitors with FOLFIRINOX regimens has shown longer survival than treatment with FOLFIRINOX regimens for pancreatic cancer patients, with reliable clinical efficacy, tolerable adverse effects, and a high safety profile.

## Figures and Tables

**Figure 1:** Comparison of serum markers (the serum marker data for this study was entered into excel software by the lead author, the statistical processing software is SPSS 25.0 for calculation, and the measurements are the mean ± standard deviation using the independent sample *t*-test. The measured values, CA15-3, CYFRA21-1, and CEA in the observation group were significantly lower than those in the reference group, and the differences were all statistically significant (*P* < 0.05). However, the CAI25 and TPS in the observation group were not significantly different from those in the reference group, and the difference was not statistically significant (*P* > 0.05).

**Figure 2:** Comparison of clinical efficacy (the count data were described by *M*(QR), and the Mann–Whitney test was used to find that 0RR and DCR were significantly higher in the observation group than in the comparison group, and all statistical tests were two-sided probability tests with a statistical significance of *P* < 0.05).

The article "Efficacy, Safety, and Impact on Patient Survival of PDL1/PD-1 Inhibitors versus FOLFIRINOX Regimens for Advanced Pancreatic Cancer" was retracted in 2023. Reasons: unreliable results or conclusions; lack of ethics approval or compliance; concerns about the data; concerns about the peer review.

**Figure 3:** Comparison of adverse reactions (the count data were described by M(QR), and the Mann–Whitney test was used to find that the patients in the observation group had hematological toxicity, neutropenia, anemia, thrombocytopenia, nonhematological toxicity, vomiting, fatigue, infection, diarrhea, The rate of adverse reactions such as intestinal obstruction and peripheral neuropathy was 10.3% lower than that of 25.8% in the comparison group, and all statistical tests were two-sided probability tests with a statistical significance of *P* < 0.05).

**Figure 4:** Survival analysis (the progression-free survival in the observation group was significantly higher than that in the comparison group, and there was a statistically significant difference between the two (*P* = 0.047)).

**Table 1:** General information [*n*, $\left(\bar{x}\pm s\right)$].

Group	Gender (male/female)	Average age (years)	Basal metabolism (kcal)	Body weight (kg)	Height (cm)
Comparison group (58)	36/22	68.78 ± 3.32	1372.34 ± 100.25	59.51 ± 10.82	159.34 ± 6.25
Observation group (58)	37/21	68.62 ± 3.66	1372.26 ± 100.64	59.57 ± 10.81	159.33 ± 6.24
*χ* ^2^/*t*	0.037	0.247	0.004	-0.030	0.009
*P*	0.848	0.806	0.997	0.976	0.993

## Data Availability

No data were used to support this study.
